The article "Utilising Induced Pluripotent Stem Cells in Neurodegenerative Disease Research: Focus on Glia" was published in 2021. Journal: Int J Mol Sci.

# Utilising Induced Pluripotent Stem Cells in Neurodegenerative Disease Research: Focus on Glia

**DOI:** 10.3390/ijms22094334

**Published:** 2021-04-21

**Authors:** Katrina Albert, Jonna Niskanen, Sara Kälvälä, Šárka Lehtonen

**Affiliations:** 1 Department of Clinical Neurosciences, University of Cambridge, Cambridge CB2 0QQ, UK; katrina.albert@gmail.com; 2 A.I. Virtanen Institute for Molecular Sciences, University of Eastern Finland, 70211 Kuopio, Finland; jonna.niskanen@uef.fi (J.N.); sarsk@student.uef.fi (S.K.); 3 Neuroscience Center, University of Helsinki, 00014 Helsinki, Finland

**Keywords:** astrocytes, microglia, oligodendrocytes, induced pluripotent stem cells, transplantation, organoids, neurodegenerative disease, humanized models

## Abstract

Induced pluripotent stem cells (iPSCs) are a self-renewable pool of cells derived from an organism’s somatic cells. These can then be programmed to other cell types, including neurons. Use of iPSCs in research has been two-fold as they have been used for human disease modelling as well as for the possibility to generate new therapies. Particularly in complex human diseases, such as neurodegenerative diseases, iPSCs can give advantages over traditional animal models in that they more accurately represent the human genome. Additionally, patient-derived cells can be modified using gene editing technology and further transplanted to the brain. Glial cells have recently become important avenues of research in the field of neurodegenerative diseases, for example, in Alzheimer’s disease and Parkinson’s disease. This review focuses on using glial cells (astrocytes, microglia, and oligodendrocytes) derived from human iPSCs in order to give a better understanding of how these cells contribute to neurodegenerative disease pathology. Using glia iPSCs in in vitro cell culture, cerebral organoids, and intracranial transplantation may give us future insight into both more accurate models and disease-modifying therapies.

## 1. Introduction

Previously only relegated to the support cells of the central nervous system, glial cells—astroglia, microglia, and oligodendrocytes—often took a back seat to neurons in terms of relative importance in neuroscience. Lately, however, researchers are discovering the central role they play in the brain, particularly when it comes to complex human disorders such as neurodegenerative diseases. With the ability to produce human glia in vitro, we have been able to study how these cells might contribute to disease aetiology and gain further insight into future therapy. Specifically, this review discusses how glial cells derived from induced pluripotent stem cells (iPSCs) are being used to better model the most common human neurodegenerative diseases, as well as a look towards how transplantation of iPSCs can work as both a model and a therapeutic strategy.

### 1.1. Glial Cells and Their Main Functions

When glial cells were first discovered they were seen only as a passive, structural cell group. These nerve adhesive cells were named glia after the Greek word meaning ´glue´ and only in further studies were the diversity and multifunctional properties of these cells unveiled. The glial cells can be divided into four major groups: 1) astrocytes, 2) microglia, 3) oligodendrocytes and 4) NG2^+^ progenitor cells (NG2, nerve/glial antigen 2). In this review, we will concentrate on the first three. The ratio of these different cell types has regional variation, but current understanding is that for each nerve cell there is approximately one glial cell, thus they make up almost half of the cells in the central nervous system (CNS) [1]. Most of the cells of the CNS have a common neuroepithelial origin [2] and in early stages of embryogenesis, these cells start to differentiate into neural progenitors. Progenitor cells then divide and differentiate first into neurons and then at a late stage of embryogenesis into oligodendrocytes and astrocytes. Microglia originate from the embryonic yolk sac and differentiate in early embryogenesis together with neurons, making them the first mature glial cells in the CNS [3,4].

Astrocytes (Figure 1) are the most abundant glial cells: depending on brain region and calculation method, the estimation is 20–60% of all the cells in the CNS [5]. Astrocytes are a diverse cell population to such an extent that, for the multiple different forms, a consensus regarding nomenclature and definitions was needed [6]. Morphologically, these cells are complex and can adjust to the changes in their surroundings [7,8,9]. They provide the structural support of the CNS and their long thin processes surround both synapses and blood vessels, creating non-overlapping territories. These contacts enable them to perform a variety of functions, including maintaining homeostasis, transferring nutrients, water, and oxygen to the neurons, and providing neurotrophic support. Astrocytes can regulate the composition and volume of the extracellular space by controlling ion concentration (e.g., Ca^2+^, K^+^), uptake of neurotransmitters, and water movement [7]. They can affect the consistency and function of the blood–brain barrier (BBB) and control the cerebral blood flow in response to neuronal activity [6]. These functions enable astrocytes to move perivascular fluids across the brain and contribute to brain waste management. This phenomenon is called the glymphatic–lymphatic fluid transport system [10,11]. It is especially effective at removing waste products during sleep [12,13], and the sleep–wake cycle is connected to astrocyte signaling [14]. The uptake and clearance of neurotransmitters (ex. GABA, glutamate) are important for the continuance of neurotransmission, and to avoid a toxic accumulation of certain transmitters [15].

The perisynaptic processes (PAPs) are thin processes of astrocytes that take part in promoting synaptogenesis and modulating the plasticity and density of synapses [7,16]. The tripartite synapse refers to communications between neurons and astrocytes, where astrocytes regulate synaptic transmission. In tripartite synaptic activity, astrocytes respond to neurotransmitters by releasing Ca^2+^, which releases gliotransmitters that, in turn, control neuronal excitability and synaptic transmission [16]. Importantly, astrocytes react to CNS damage from pathological processes such as neuroinflammation, trauma, and ischemia through reactive astrogliosis [6,7,17]. 

In reactive astrogliosis, astrocytes go through biochemical, morphological, metabolic, and physiological changes, resulting in gain of new functions or modulations in the existing homeostatic ones [6]. Astrocytes upregulate the expression of glial fibrillary acidic protein (GFAP), vimentin, and nestin [17]. The cellular processes become shriveled, and the astrocytes change their excretion of proteases, cytokines, and growth factors. Depending on the magnitude of the astrogliosis, it can lead to the formation of a glial scar from substantially proliferating astrocytes. In mild astrogliosis, the cells do not proliferate but rather alter their gene expression.

Microglia (Figure 1) make up approximately 5–10% of the cells of the CNS. They are resident macrophages that provide immunosurveillance to the CNS [18]. They are the first glial cells present in the developing brain and have a fundamental role in early development [19]. During synapse maturation, microglia take part in synaptic pruning when the turnover is the highest [20]. They also rigorously survey the myelinated tracts during development [21]. To give an idea of the mobility of these cells, a recent study observed microglia visiting myelinating oligodendrocyte regions roughly every four hours. They engulf myelin sheaths but not the oligodendrocytes themselves. Microglia are plastic and quickly respond to their surroundings by, e.g., changing morphology from ramified—resting or surveilling state—to ameboid, an activated state [22]. The ramified microglia have round cell bodies with only a small cytoplasmic area and extensive branching processes. If there are any pathological signals/molecules or abnormal signaling—or indeed no signals—coming from the other surrounding CNS cells, the microglia turn into an amoeboid, activated state, where the branches morph into thick pseudopodia.

Activated microglia are extremely mobile and move quickly towards the area of interest, where they can release cytotoxic substances and undergo phagocytosis together with manifesting anti-or pro-inflammatory responses. For example, they can engulf α-synuclein released from neurons which may prevent neurodegeneration [23]. α-synuclein is a presynaptic protein with a suggested role in neurotransmitter release in the healthy brain and a strong relationship with several neurodegenerative diseases (e.g., Parkinson’s disease (PD) and Alzheimer’s disease (AD)) [24,25,26]. In recent studies, microglia have also been observed to play a role in maintaining neural circuit connectivity in the adult brain, where an in vivo test with mice showed that depleting microglia increased neural circuit connectivity [27].

Oligodendrocytes make up approximately 20–75% of the cells in the CNS, depending on the region [5], and they are most numerous in the white matter. Myelin production is the primary role of oligodendrocytes (Figure 1) [28]. The myelin sheath wraps around axons, improving neural conductivity. The myelin sheath is not a static structure as de- and remyelination sculpts the circuits forming memories and enabling learning [28,29]. However, the role of oligodendrocytes is not limited to myelin production, they also take part in supporting, modulating, and regulating neurons. They give axons metabolic support by expressing monocarboxylic acid transporter 1 (MCT1), a glycolytic substrate transporter that functions as a major supplier of lactate to axons and neurons [30]. Oligodendrocytes produce factors that promote neuronal survival and increase axon length (e.g., glial cell-derived neurotrophic factor, GDNF) [31]. They also inhibit neurite growth and stabilize neuronal connectivity. Oligodendrocytes also respond to oxygen levels in the brain through hypoxia-inducible factor (HIF) signaling and drive angiogenesis in the white matter [32].

### 1.2. Induced Pluripotent Stem Cells (iPSCs) to Generate Glia

The cells to produce iPSCs can be harvested from any source, but they will only model the organism they have been harvested from [33,34,35]. To study human diseases, human iPSCs are required since, despite some evolutionarily conserved similarities, rodent and human brains differ from each other [36]. Human iPSCs are obtained from human somatic cells which can be taken from, for example, a skin biopsy. This, therefore, bypasses some of the ethical issues associated with utilizing human tissue for research purposes. The differentiated somatic cells can be reprogrammed back into pluripotency through various different methods [37,38]. In the most classical method, pluripotency genes—so-called Yamanaka factors (Oct3/4, Sox2, c-Myc, and Klf4)—are introduced into adult fibroblasts through retroviral transduction [38]. Currently, the most commonly used method to generate iPSCs is via the non-integrating Sendai viral vector [39]. There have also been many advances in iPSC generation and methods such as epigenetic regulation, microRNA manipulation, and nonviral methods have arisen in recent years [40,41]. iPSCs can be differentiated into various cell types, including neurons and glia, making them a powerful tool to study human CNS cells in vitro (Figure 2). As will be discussed further below, iPSCs have been successfully differentiated into astrocytes [42,43,44], microglia [45,46], and oligodendrocytes [47,48,49,50,51] from both healthy subjects and patients. This process can then be harnessed to study how these cells and their factors may contribute to disease in a human-specific way, both in vitro and via transplantation in vivo.

In general, there are no disease-modifying therapies for complex human disorders. Therefore, understanding mechanisms has been paramount in moving this research further. The ability to generate iPSC-derived glia, combined with our increasing understanding of glia involvement in human disease, can give us insight into understanding these conditions in order to find cures. In addition to neurodegenerative diseases, neuropsychiatric disorders are prime candidates for the use of iPSCs to study mechanisms. Similar to neurodegenerative iPSC research, neuropsychiatric disorders have mainly used neurons derived from patients, but recent studies have begun to use patient-derived iPSC glial cells as well (reviewed in [52]). For example, astrocytes derived from Alexander disease patients, cultured together with oligodendrocyte progenitor cells (also patient-derived), decreased the number of these progenitor cells and led to fewer myelinating oligodendrocytes—a main pathological hallmark of the disease [53]. Researchers using microglia and isolated synaptosomes derived from schizophrenic patients found increased engulfment of the synapses by the microglia compared to healthy control-derived cells [54]. This was considered to mimic the increased synaptic pruning present in postmortem schizophrenic patient brains. Along with using iPSC-derived glial cells to directly model these disorders, these cells can be a useful source for gene expression analysis in order to elucidate involvement of genes in human-specific conditions. A study using astrocytes derived from the skin fibroblasts of violent offenders showed upregulation of genes already associated with autism [55]. Studies such as this can give researchers a better understanding of which genes could be involved in multifaceted human diseases.

It is clear that glia play a role in neuropsychiatric disorders and using patient-derived cells more closely resembles the human condition. Additionally, glial cells are also heavily implicated in neurodegenerative disease mechanism and using patient-derived iPSCs to model these diseases is an important avenue of research, discussed in detail below.

## 2. Glia involvement in Neurodegenerative Diseases

Neurodegenerative diseases are an assortment of different disorders that are associated with neuronal loss, cellular dysfunction, and pathological accumulation of proteins in the brain. The symptoms of these diseases vary from motor to cognitive dysfunction. All of the diseases listed below have evidence of glial cell involvement in the onset and progression (Table 1). Many studies have observed neuroinflammation, reactive microglia and astrocytes, as well as oligodendrocyte dysfunction in the patient brain. Using cells harvested from patients with causative mutations, iPSC models can recapitulate the key aspects of these diseases. Though studies utilizing glial cells derived from iPSCs are only recently emerging.

AD is the leading cause of dementia worldwide (Table 1) and human iPSC-derived cells have been used extensively to study aspects of the disease in vitro. Disease-associated AD astrocytes have been identified from single-nucleus RNA sequencing (snRNA-seq) [57], where, e.g., massive gliosis was observed upon AD initiation. Astrocytes derived from iPSCs from AD patients with the *PSEN1 ΔE9* mutation, manifest with increased amyloid-β (Aβ) production and oxidative stress [60], altered metabolism of fatty acids [99] and Ca^2+^ [60], together with reduction in lactate secretion [60]. The iPSC *PSEN1 ΔE9* AD astrocytes use less glycolysis for energy production and were much more oxidative than the control cells, thus elevating the levels of intracellular oxygen species that are toxic to neurons [60]. iPSC-derived AD microglia, generated from patients with either sporadic AD [63] or isogenic lines from healthy donors with risk gene *APOEε4* edited with CRISPR/Cas9 [100], are more immunoreactive compared to control cells. This finding is supported by snRNA-seq data from human AD brains and non-demented control brains [57,62]. They display altered phagocytosis (e.g., elevated general (sporadic AD model) [63] or impaired Aβ phagocytosis (*APOEε4*) [100]), and upon lipopolysaccharide (LPS) treatment, enhanced cytokine production (IL-6, IL-10, TNF-α, IFN-γ [63]). iPSC-derived oligodendrocytes have not yet been used to model AD, although changes in the oligodendrocyte differentiation and myelination have been associated with the disease, and several AD risk genes have important roles in oligodendrocyte biology [59,64]. For example, decreased myelination, reduced oligodendrocyte size, and death of oligodendrocytes have been depicted both in postmortem AD brain and in vivo mouse studies [64].

The molecular mechanisms behind amyotrophic lateral sclerosis (ALS) (Table 1) are still somewhat unknown, but the non-cell autonomous processes are becoming more evident. Reactive astrocytes have been identified surrounding the degenerating motor neurons in ALS [17]. iPSC-derived astrocytes from ALS patients carrying the G4C2 repeat expansion in the *C9orf72* gene, cultured together with motor neurons, cause motor neurons to lose their excitability and action potential output [66], where astrocyte dysfunction precedes these motor neuron perturbations. A mutation in the *C9orf72* gene is common for both ALS and frontotemporal dementia. Astrocytes contribute to the neurotoxicity by excreting toxic factors such as effectors of necroptosis, reactive oxygen species, proinflammatory cytokines and inflammatory mediators [17,66]. ALS also manifests with progressive microgliosis, and microglial dysfunction appears to be one of the earliest occurrences in disease progression [65]. Microglial dysfunction is proximal to motor neurons and precedes symptom onset and astroglial dysfunction. Using iPSC-derived microglia-like cells, derived from patients with the *C9orf72* genetic mutation, the cells show increased inflammatory responses, and upon Aβ or synaptoneurosome exposure, disturbed phagocytosis [68]. The oligodendrocyte progenitor cells, NG2^+^ cells, are wildly proliferating at the end stage of ALS, with the proliferation rate growing 20-fold; however, this oligodendrogenesis does not lead to oligodendrocyte accumulation [69]. In terms of neurodegeneration in ALS, oligodendrocytes contribute to motor neuron death by excreting soluble neurotoxic factors and through cell-to-cell contacts [70]. A significant decrease in motor neuron survival was observed 4 days after they were grown in ALS-oligodendrocyte conditioned media. When growing iPSC-derived ALS oligodendrocytes, from patient iPSCs with sporadic ALS or ALS with a *SOD1D90A, TDP43G298S, C9ORF72*, or *FIG4C27T* mutation, together with healthy motor neurons, 72 hours post plating the motor neurons started to manifest with an axonal beading phenotype and the cell survival decreased by 50–60%. Additionally, ALS oligodendrocyte lactate production starts to reduce at three weeks post plating—they produce less lactate overall compared to control and express lower levels of MCT1 transcript, both features that are important to neuronal energy metabolism. 

One of the most well-known prion diseases is Creutzfeld–Jacob disease (CJD) (Table 1), where there is evidence of both reactive astrocytes and microglia [71,75]. In CJD, astrocytes have a complex role and the reactive state has a distinct phenotype from other neurodegenerative diseases [71]. Interestingly, the reactive astrocytes appear to have disease progression delaying properties, where disabling the astrocyte morphosis to a reactive state accelerated the disease progression and resulted in early microglial dysfunction [71]. According to findings made from studies performed with iPSC-derived astrocytes (cells from healthy donors), the cellular susceptibility to prion infection is dependent on an appropriate CNS cellular phenotype [76]: astrocytes accumulate prion proteins when the CJD inoculum and cell *PRNP* codon 129 genotype matches. There are also peculiar findings in relation to astrocyte and oligodendrocyte interactions associated with CJD, when the disease progresses to a more severe state, the reactive astrocytes engulf oligodendrocytes in a process called emperipolesis [72,74]. Evidence of glial cell association with CJD has been found [75] but to date not many studies have been performed with iPSCs.

Huntington’s disease (HD) (Table 1) is a hereditary neurodegenerative disease. The HD astrocytes appear to progressively lose their normal functions as mutant huntingtin protein accumulates [78]. Several observations have been made using iPSCs: iPSC-derived HD astrocytes (iPSCs derived from patients with *HTT* mutations) fail to support maturation of iPSC neurons as well as the control astrocytes [80], neuronal electrophysiological activity is dampened in HD astrocyte-control neuron co-cultures as a result of impaired Ca^2+^ modulation, and these HD astrocytes are unable to protect the neurons against glutamate-mediated toxicity. Previous studies have found that glutamate transporters are downregulated in HD astrocytes, and this impairs the natural glutamate uptake via astrocytes which disrupts the normal neurotransmission and has neurotoxic effects [15]. The HD astrocytes are essentially reactive astrocytes. Recent studies have indicated that microglial activation precedes astrocyte activation, showing that microglia also play a key role in HD onset and progression [15,56,79]. White matter alterations have been documented in HD human and mice studies together with oligodendrocyte dysfunction and impaired remyelination [82,83,84]. However, in general, HD has not been extensively studied using iPSC-derived glial cells, as the main focus has been on the iPSC-derived neuronal cells [101].

PD is the second most common neurodegenerative disorder (Table 1). Neuroinflammation is seen as one of the key features of PD [56,85,86]. Indeed, iPSC-derived astrocytes (from patients with the *LRRK2* G2019S mutation) morph into reactive astrocytes after an inflammatory stimulus and respond with a stronger inflammatory response compared to control, e.g., by releasing more proinflammatory cytokines [87]. These PD astrocytes also have disturbances in metabolism, mitochondrial function and respiration, loss of neurotrophic factor secretion, downregulation of glutamate intake, and disturbances in Ca^2+^ homeostasis [87,102]. iPSC *LRRK2* G2019S astrocytes upregulate the expression of α-synuclein [87], a presynaptic protein of which aggregates form Lewy bodies in PD [24,25]. Control neurons cultured together with PD *LRRK2* G2019S astrocytes start to show signs of neurodegeneration—similar to the ALS co-culture studies—and accumulate α-synuclein [102]. In PD, the microglia lose some of their beneficial physiological functions and gain detrimental inflammatory functions [88]. It was shown that iPSC-derived *LRRK2* G2019S microglia are more immunoreactive than the controls (isogenic or healthy) [89]. When an immune stimulus was given (IFN-γ or LPS), the PD microglia decreased their motility but increased their phagocytosis and metabolic activity. These PD microglia were also seen to have defects in the transcription factor NF-κB p65 nuclear translocation. NF-κB p65 plays a key role in processes such as cell survival, inflammation, immunity, differentiation, and apoptosis. When applying iPSC-derived *LRRK2* G2019S PD microglia conditioned media to neurons, clear signs of an inflammatory environment were seen and neurite elongation was affected [89]. Early involvement of oligodendrocytes in the onset of PD has been suggested in genome wide association studies [91], but studies using iPSC-derived oligodendrocytes are lacking.

Spinocerebellar ataxias (SCAs) (Table 1) are a collection of neurodegenerative diseases. Most of the hereditary SCAs are characterized by abnormal expansion in the sequence coding polyglutamine (polyQ) peptides and by the polyQ aggregates in the cerebellum [93,103]. There is evidence of early astrocyte and microglia activation in SCA1 [92], which can be seen in the increased levels of proinflammatory cytokines IL-6, TNFα, and MCP-1. Glutamate-treated neurons, derived from iPSCs from patients with SCA2 and SCA3, downregulate the glutamate receptor genes and dysregulate intracellular Ca^2+^ [93]. The studies in vivo from SCA7 mice suggest a link to Bergmann glia, protoplasmic astrocytes in the cerebellum, that produce neurodegeneration by impairing glutamate transport [104]. In a SCA3 mouse model, oligodendrocytes show early transcriptional changes, toxic gain-of-function mutations, and demyelination [94]. The implementation of iPSC models to study SCA has not been fully utilized and the findings regarding glial involvement with these diseases have mostly been done with in vivo rodent models [92,94,104,105].

Loss or functional inactivation of the gene survival motor neuron 1 (*SMN1*) causes spinal muscular atrophy (SMA) (Table 1). The disease phenotype is considered as non-motor neuron-autonomous and strong glia involvement has been observed as well as general neuroinflammation, where proinflammatory cytokines secreted by both astrocytes and microglia are elevated (IL-6, IL-1β, TNFα) [95,96]. Astrocytes have been seen to contribute to the pathogenesis of SMA in particular [95]. The iPSC-derived SMA (from patients with *SMN2* or *SMN1*) astrocytes manifest with morphological and cellular changes that can be observed prior to onset of motor neuron loss [106]. They have disrupted Ca^2+^ signaling where the basal Ca^2+^ is significantly increased but the Ca^2+^ response to ATP significantly decreased compared to control. The ERK1/2 pathway, which can lead to apoptosis when activated by Ca^2+^, is upregulated in iPSC-derived *SMN1/SMN2* SMA astrocytes [106]. These astrocytes express low levels of SMN protein and have significantly shorter cellular processes [95,106]; low levels of SMN protein lead to progressive astrocyte activation (evidenced by expression of markers for reactive astrocytes (GFAP and vimentin)). The SMA iPSC astrocyte cultures also produced and secreted less GDNF than control iPSC astrocyte cultures [106]. Without GDNF, astrocytes fail to promote the survival of spinal motor neurons leading to apoptosis. Most microglia and oligodendrocyte associated SMA studies have been done using in vitro models [96]. The microglia have been seen to obtain a more proinflammatory morphology and have enhanced phagocytosis, leading to a process called synaptic stripping. In terms of oligodendrocyte involvement, myelin basic protein (MBP) and NG2 expression were found to be lower in the spinal cords of *SMNΔ7* mice compared to control [98]. NG2 expression is essential for oligodendrocyte differentiation and proliferation of the oligodendrocyte progenitor cells. This phenomenon was also reported to occur prior to motor neuron degeneration: the cells with low NG2 expression levels had high Notch expression, as the low levels of NG2 failed to inhibit Notch activation. Notch signaling is a master regulator of neural development. When activated, it disrupts the precursor cell differentiation to myelinating oligodendrocytes, but it also affects the differentiation and proliferation of astrocytes [107].

The above neurodegenerative diseases have glial dysfunction followed by death of neurons in common. In many studies, the neuronal damage is traced back to an inflammatory microenvironment where reactive astrocytes are one of the main causes of this damage. Microglia are in a constant surveillance state and quickly react to their surroundings. According to prior studies, reactive microglia are needed to induce reactive astrocytes [56]. Reactive astrocytes lose their ability to uphold neuronal survival and outgrowth, lose their synaptogenesis and phagocytosis ability, and become powerfully neurotoxic. This reactive state then induces neuron and oligodendrocyte death. Reactive astrocytes have a high expression of complement component C3. In a recent study, to visualise the reactive C3 positive astrocytes in different neurodegenerative diseases, in situ hybridization and immunochemistry were performed on postmortem tissue from patients with AD, ALS, HD, multiple sclerosis (MS), and PD. Reactive astrocyte markers GFAP, S100β, and C3 labeled positive astrocytes were found in regions traditionally associated with the respective diseases, and further qPCR analysis confirmed this finding.

## 3. 3D Brain Organoids as Models of Neurodegenerative Disease

A major barrier which hinders the study of neurodegenerative diseases is the inaccessibility of relevant biological material: human brain tissue. Early research was restricted to histological samples obtained postmortem from symptomatic patients and healthy controls [108]. However, neurodegenerative diseases are progressive in nature: pathological changes in the brain can occur decades before the onset of clinical symptoms, diagnosis by a physician, and death [109,110,111,112]. While advances in biomedical imaging have expanded our ability to study the brain in living subjects [112,113], brain biopsy remains an invasive and high risk procedure. Thus, brain tissue samples from living patients continue to remain extremely limited. For this reason, developing disease models that facilitate observation and sample collection throughout the course of the disease—from onset to advanced pathology—is key to elucidating the degenerative processes underlying these diseases. They are also critical for exploration and evaluation of potential treatments and medications. 

Due to the difficulty of studying the molecular biology of neurodegenerative diseases in living patients, much effort has been put into developing animal models for studying disease pathology and for evaluating drug candidates. However, developing preclinical models of the two most prevalent neurodegenerative diseases, AD and PD, has proved especially challenging [114]. Preclinical models of AD have proved to be unreliable predictors of therapeutic effectiveness in human subjects, and drug candidates for AD have an exceptionally high failure rate of 99.6% in clinical trials [115]. This indicates a desperate need for improved disease models which are capable of more accurately representing the disease biology in humans. Creation of iPSCs has revolutionized in vitro study of human disease by granting access to a virtually unlimited supply of human cells. However, conventional 2D cell cultures cannot recreate the intricate cell architecture and microenvironment of human brain tissue.

Cerebral organoids derived from iPSCs, first described by Lancaster et al. [116], have shown potential to overcome the inaccessibility of human brain tissue (Figure 3). The cerebral organoids generated by Lancaster et al. contain a variety of brain regional identities and display the characteristic layering of progenitors, precursor cells, and neurons seen in the developing human brain. Brain organoids are a promising novel platform for compound screening applications, as they can be produced in large quantities sufficient for high-throughput experiments. However, heterogeneity and random occurrence of different brain regions in cerebral organoids limit their utility as robust disease models [116]. To address this issue, various strategies for guiding the development of the organoid tissue towards a specific regional fate have been developed [117,118,119,120,121]. Heterogeneity will remain an issue for “handmade” organoids, as manual pipetting and handling will introduce variability within and between organoid batches. For experiments requiring highly homogenous samples, fully automated processes that minimize human error and batch effect are desired [122]. Optimization of differentiation conditions and automation, while still very active areas of research, have led to the creation of more homogenous, brain region-specific organoids capable of recapitulating key molecular hallmarks of neurodegenerative diseases.

In addition to neurons, brain organoids give rise to both astrocytes and oligodendrocytes [118,121,123,124,125]. As discussed, glial cells—the caretakers of the CNS—are increasingly recognized as key contributors to neurodegenerative diseases (Table 1). The co-occurrence of neurons and glia in brain organoids makes them an attractive model for studying the non-cell autonomous mechanisms of neurodegeneration. However, microglia are inherently absent in brain organoids induced with dual-SMAD inhibition, which directs the iPSCs towards a neuroectodermal fate. This inhibits the emergence of microglia progenitors, which originate from the mesodermal lineage and migrate from the embryonal yolk sac to the brain [126]. Brain organoids also lack endothelial cells and thus are not vascularized. To “complete” the brain organoid model, separately differentiated endothelial cells, microglia-like cells or mesodermal progenitors must be integrated into the organoid. Interestingly, functional microglia-like cells expressing Iba1 have been reported to occur spontaneously in brain organoids generated without SMAD inhibitors [127]. During brain development, microglia are known to modulate synaptic remodelling and have been shown to promote functional maturation of neurons and cortical networks in cerebral organoids [128,129]. Transplanted microglia exhibit chemotactic attraction towards neuronal tissue, followed by migration and extension of processes resembling the ramified (“surveillant”) microglia present in the CNS. Upon injury, organoid-resident microglia assume ameboid morphology and migrate towards the injured site, demonstrating in vivo-like functionality [45]. Attempts at creating vascularized organoids have relied on in vivo transplantation and invasion of host vessels into the organoid [130,131], but this is not ideal as patient iPSC-derived vessels are more desirable. Pham et al. [132], have reported successful integration of endothelial cells into organoids, while Wörsdörfer et al. [133] generated vascularized organoids with Iba1+ microglia by introducing mesodermal progenitors. In addition, Cakir et al. [134] demonstrated perfusion of blood vessels generated via induced *ETV2* expression. The addition of functional vasculature in brain organoids could overcome two significant issues: firstly, providing perfusion throughout the organoid could prevent necrotic cores, which are a pervasive problem in larger organoids. Secondly, functional coupling between vessels, astrocytes, and neurons could serve as an excellent platform for modeling BBB function and the neurovascular unit. 

Remarkably, cerebral organoids derived from iPSCs of a patient with familial AD (fAD) have been observed to replicate key pathological hallmarks of AD, such as formation of Aβ aggregates, hyperphosphorylated tau, and increased apoptosis. It is especially notable that AD pathology emerges organically in patient-derived organoids without the need to induce overexpression of fAD genes [135,136,137]. Raja and colleagues noted that Aβ pathology precedes tau aggregation in organoids. Their findings were consistent across multiple fAD iPSC lines and AD pathology was ameliorated by treatment with γ-secretase and BACE1 inhibitors. It is likely that the 3-dimensional (3D) extracellular space present in organoid cultures facilitates concentration and subsequent aggregation of plaque-forming proteins [135,138]. The ability of cerebral organoids to form mature neuronal networks enables interrogation of functional defects in fAD. *PSEN1/2* and *APP* fAD organoids display asynchronous calcium transients, increased neuronal activity and hyperexcitability [137,139]. Presence of the *APOEε4* allele is the most notable genetic risk factor for sporadic AD, but the exact molecular mechanism behind this remains elusive. In contrast to fAD organoids, in which pathology arises relatively early, Lin et al. [100] report delayed emergence of AD pathology in brain organoids harboring the *APOεE4* allele. This also provides evidence for the involvement of astrocytes in sporadic AD, which is further corroborated by reduced Aβ uptake and cholesterol accumulation in *APOEε4* astrocytes. Zhao et al. [140] have reported a similar increase in phospho-tau load in *APOEε4* organoids compared to *APOEε3* organoids, where increased phospho-tau was already evident in four-week-old AD and *APOEε4* organoids.

Midbrain organoids (MOs) are an attractive model for PD. Organoids patterned towards the midbrain are enriched in dopamine (DA) neurons, which are functionally mature and express midbrain-specific markers such as EN1, FOXA2, LMX1A, and TH [121,141,142]. Neuromelanin inclusions characteristic of the human *substantia nigra pars compacta* have been observed after two months in culture [141]. MO DA neurons have been shown to be susceptible to neuronal death caused by the known neurotoxins 6-hydroxydopamine (6-OHDA) and 1-methyl-4-phenyl-1,2,3,6-tetrahydropyridine (MPTP) [118,123,143]. MOs derived from iPSCs carrying the known PD risk mutation *LRRK2*-G2019S have been shown to demonstrate aberrant accumulation and deposition of α-synuclein, which was successfully ameliorated by LRRK2 kinase inhibitor treatment [123]. MOs derived from a patient with idiopathic PD (iPD) also replicate molecular features of the disease: Chlebanowska et al. [144] found significantly reduced TH expression in iPD MOs compared to healthy controls. TH expression in iPD MOs plateaued at 27 days and decreased at later time points, whereas increasing levels of TH were observed in healthy MOs throughout the experiment. In addition, expression of early midbrain neuronal markers FOXA2 and LMX1A were markedly lower in iPD MOs. 

Cerebral organoids exhibit similar developmental events as the fetal human brain [116,125,145,146,147], which indicates that they could be excellent models for neurodevelopmental disorders. Principal component analysis by Jo et al. [141] of gene expression in generated MOs, prenatal midbrain, and adult midbrain indicated that MOs are more prenatal midbrain-like than adult midbrain-like. In contrast, the most common neurodegenerative diseases, AD and PD, are highly prevalent in the elderly population. Recapitulating the ageing brain in an inherently immature organoid is a challenge which may limit their usefulness as models of advanced neurodegenerative diseases. Strategies for inducing ageing-like effects in iPSC-derived neurons via oxidative stress [148,149] or overexpression of progerin [150] have been described. Somewhat surprisingly, the immature nature of cerebral organoids has provided valuable insight into dysfunctions of neurogenesis in AD. It appears that mutant *PSEN1* expedites neuronal differentiation by reducing Notch signaling, which results in diminished populations of neural progenitor cells in fAD organoids [151]. Premature neuronal differentiation and subsequent progenitor depletion has also been observed in sporadic AD organoids [152]. In addition, Meyer and colleagues provided evidence that *APOEε4* induces dysregulation of the transcriptional repressor REST, leading to upregulation of neuronal differentiation genes in sporadic AD neural progenitors. Similarly, *PINK1* knockout MOs display reduced numbers of Tuj1/TH double positive cells but no reduction in Tuj1+ cells compared to control MOs, indicative of impaired DA neuron differentiation [153]. Mutations in *PINK1* have been associated with early-onset PD. The curious connection between impaired neurogenesis and onset of neurodegenerative disease warrants further investigation. 

Cerebral organoids derived from iPSCs are a promising way forward for studying neurodegenerative diseases, where instead of a single cell population in the culture dish, something more akin to the whole brain environment is achieved. This is a useful strategy to model human disease more accurately in vitro. Additionally, the ability to test exogenous material on these models and how it may contribute to disease state, as well as transplanting these organoids to animals, are important avenues of future research.

## 4. In Vivo Transplantation of iPSCs in Neurodegenerative Diseases

More than 40 years ago, researchers transplanted human fetal tissue to rodent [154,155] and non-human primate [156,157] PD models, resulting in fetal DA cells surviving in the brains of these animals and behavioural improvements. This led to clinical trials in Parkinson’s patients where injection of embryonic DA cells to the putamen of patients survived, reinnervated the striatum, and resulted in symptom benefit in several recipients [158,159,160]. Despite only modest improvement in some patients and the presence of Lewy bodies (α-synuclein rich pathological hallmark of PD [25]) in grafted neurons [161,162], survival and integration of these cells to the human brain demonstrate a strong positive outcome from these trials. As such, there are currently ongoing trials using embryonic stem cells in PD (preclinical study of one ongoing trial [163]), although this review will focus further on iPSC studies. With the advent of iPSCs, research on potential therapies as well as human disease modelling shows great promise going forward.

Having a readily available and replenishable pool of cells that can be differentiated into various cell types without the ethical issues associated with using human fetal tissue continues to be a powerful tool to model disease and test drugs on. Along with PD, several lines of research have aimed to replace dead or damaged cells in the respective rodent model of disease in order to bring a stem cell-based disease-modifying therapy to the clinic. For example, transplantation of human iPSCs differentiated to neural stem cells in rodent models of spinal cord injury [164,165,166] and ischemic stroke [167,168,169] have been successful. These cells survive, differentiate, migrate, and result in functional recovery in some cases. However, not all studies have demonstrated positive results [170]; a study of wild-type mice with spinal cord injury and receiving immunosuppression therapy did not show long-term survival of the cells and there was no evidence of functional recovery in the model. This demonstrates the need for both longer follow-up times as well as using conditions that more closely mimic how a real-world therapy would be carried out. Additionally, of high concern in the field of stem cells in general has been the issue of tumorgenicity once they are transplanted to the target organ. As such, it has been shown that transplantation of undifferentiated iPSCs can result in tumorigenic outcomes [171,172]. Therefore, the step to differentiate these cells to neural stem cells or progenitors before injecting them into the brain is a critical step in the process.

In addition to the above-mentioned brain diseases, neurodegenerative diseases are potential candidates for stem cell transplants. As alluded to above, PD is the furthest along in this regard. IPSCs derived from human patients were first differentiated to DA neurons and then successfully transplanted to a rat model of PD where they survived, began to grow axons, and led to functional recovery [173] (Table 2). It was also demonstrated that iPSCs derived from idiopathic patients versus healthy individuals did not differ in their ability to survive and function in the rat brain, indicating that a patient’s own cells could be used to differentiate and transplant [174]. Human iPSC transplant has been successful in a non-human primate model of PD [175] and, last year, a study was published with a human patient [176]. In the human case, cells were derived from the patient, differentiated to DA neuron progenitors, and transplanted to the putamen without immunosuppression. The cells seemed to survive and result in some functional recovery—although the long-term outcome remains to be seen. The implications of using a patient’s own cells could be incredibly important going forward, as there would be no need for immunosuppression and less concern of rejection. However, cells will still need to undergo strict good manufacturing practice and testing. There are currently ongoing clinical trials using iPSCs for Parkinsonian patients [177,178].

Along with PD, there have been successful transplants of iPSCs as therapy in rodent models of AD, ALS, and HD (Table 2). Transgenic mice used to model AD via overexpression of the familial *APP* mutation [187] were transplanted with neuronal precursors to be differentiated into cholinergic neurons that were derived from human iPSCs [179]. The cells, injected bilaterally to the mouse hippocampus, developed into cholinergic neurons that survived and improved spatial memory compared to the transgenic mice that did not receive the transplants. In ALS, transgenic rats carrying the human *SOD1*(G93A) mutation (associated with a familial form of ALS [188]) were transplanted with neural progenitor cells to the spinal cord which resulted in the majority of progenitors differentiating to mature neurons at 60 days. Some of these cells began to resemble motor neurons in their morphology [189]. In terms of a possible therapeutic application, another study using the SOD1 mouse model used both intrathecal and systemic administration of human iPSCs as opposed to intracranial or spinal cord injection [180]. The authors differentiated cells to neural stem cells that were preferentially selected for factors enabling them to cross the BBB. Transgenic mice had neural stem cells present in the spinal cord in both administration paradigms, whereas the wild-type did not—the authors hypothesized that the BBB is more permeable in this model. Importantly, the mice had improvement in motor behaviour, extended survival, reduced gliosis, and an increase in number of motor neurons compared to the vehicle treatment. This study gives proof-of-concept to less invasive procedures for transplanting iPSCs which avoids potentially complicated brain surgery, particularly in conditions where the BBB may be compromised (ex. stroke). In addition to AD and ALS, iPSCs have shown success in HD. iPSCs derived from a juvenile HD patient were differentiated to neural precursor cells and injected into the striatum of quinolinic acid lesioned rats (toxin model of HD) [182]. Behavioural improvements were observed in the rats as well as mature neurons in the striatum, some of which developed a GABAergic phenotype. The authors observed that the differentiated neurons in culture did not form aggregates, nor did the rats at the conclusion of the experiment (12 weeks post-transplantation). However, when the authors examined a separate cohort of wild-type, non-lesioned mice at 33 and 40 weeks post-transplantation, they found aggregate pathology. The authors speculated that this finding could be due to the longer time period the cells were in the brain versus in the culture dish, as neurodegenerative diseases develop over long timescales (years, instead of days or weeks). Along with this, it could be that the whole brain environment of an organism incurs differential effects on aggregation outcome. These results should be taken into account when developing a potential therapy: iPSCs in the dish do not mimic timescale or brain-environment interactions when it comes to aggregate formation and consideration needs to be taken about the source of cells used for derivation. This may put a damper on the use of autologous cells from a patient for therapy, unless they are first tested in vivo at further time points and/or have been edited for mutations (ex. by using CRISPR technology).

It should be emphasized that the above transplant studies use human iPSCs in animal models, but there have also been studies with iPSCs derived from rodents and transferred to rodents, such as in traumatic brain injury [190,191], SMA [192], and HD [193,194]. The former is likely more clinically relevant, however, both in terms of therapy and modelling disease.

While iPSCs are a promising avenue for replacing neurons in neurodegenerative diseases, finding a disease-modifying therapy for these complex disorders is a difficult endeavour. Using animals to model multifaceted human diseases that generally do not develop naturally in them and incorporate a wide variety of pathological events and outcomes, is at best complicated and at worst futile. As mentioned above, it is well-known that drugs tested in animal models of human brain diseases often fail in the clinic [195,196,197,198] and this is related to issues of reproducibility and validity of the models [199,200,201]. In other words, whether the model you are using is working in different labs with minor modifications, and whether the model is truly reporting what you say it is. Having a robust and consistent protocol that is not prone to small changes (ex. different equipment used) and is fully and accurately reported in the literature are ways of ensuring reproducibility between labs. Model validity depends highly on outcome measures, for example, researchers must be careful when translating rodent physiology to humans. These are some of the important aspects of translational research to focus on when using animals to model human disease. One direction the field of neurodegenerative diseases is taking relates to utilising iPSCs to model disease in 2D and 3D cell culture as detailed above. The next step is then using these human iPSCs to model neurodegenerative diseases in rodents (Figure 4) in order to achieve a “humanized” model—a model that more closely resembles the human condition.

To date, the most work towards a humanized model of neurodegenerative disease using iPSC transplants has been done in AD, where human iPSCs are transplanted to transgenic mice to create a chimeric human-mouse model. In the first published study of its kind, the authors differentiated human iPSCs into cortical precursors and transplanted them to wild-type or transgenic neonatal mice [183]. The transgenic mice expressed human AD mutations *APP* as well as presenilin 1 (*PSEN1*) [202] and were crossed with immunodeficient mice to facilitate the graft. The progenitors differentiated to cortical neurons and integrated to the mouse brain as well as showed the presence of Aβ plaques. Interestingly, along with the transgenic mouse host tissue, the human neurons showed clear signs of AD pathology: neuroinflammation around the plaques and dystrophic neurites at 4 months post-transplantation, and pathological forms of tau at 8 months post-transplantation. Additionally, in contrast to the mouse host tissue, the transplanted neurons had changes in synaptic markers at 4 months and showed neuron loss at 6 months post-transplantation. Finally, the authors showed that the transplanted human neurons take on a similar transcriptomic profile to human AD brain samples. Taken together, these results indicate that the differentiated iPSCs transplanted to the transgenic mouse model may recapitulate the features of AD in humans in contrast to using the mouse alone to model the disease. In another study [184], the iPSCs were generated from isogenic *APOEε3/3* and *APOEε4/4* lines, genetic variants that can confer a low or high risk to develop AD, respectively [203]. These cells were then differentiated in to neurons and transplanted to the hippocampi of both transgenic mouse lines with human *APOEε3* or *APOEε4* knocked in (7-month-old mice). Along with survival and functional integration of the neurons in the mice, the authors showed that *APOEε4/4* neurons transplanted to *APOEε4* mice had gene transcriptional profiles indicating synaptic dysfunction and dysregulated calcium homeostasis, and these neurons produced more Aβ aggregates compared to the neurons transplanted to the *APOEε3* mice. An additional interesting finding from the study was that the microglia of the *APOEε4* mice showed fewer Aβ aggregates from both the *APOEε3/3* and *APOEε4/4* neurons. This could indicate that the endogenous microglia in the mice with the AD-prone mutation are less efficient at taking up human-derived aggregates.

As it has become increasingly clear that glial cells, along with neurons, play an equally central role in neurodegenerative diseases (Table 1), and that brain environment is important for how differentiated and transplanted iPSCs function in vivo, recent studies have looked at transplanting glial progenitors to the rodent brain. Previous studies have shown that iPSCs can not only be differentiated into neuronal progenitors, but specifically glial cells as well. Human iPSCs that were differentiated into oligodendrocyte progenitors and transplanted to the mouse brain resulted in both oligodendrocytes and astrocytes that were integrated, functional, and successfully rescued a model of congenital hypomyelination [204]. In another ALS study using the mouse SOD1 model, the authors transplanted neural stem cells that were rich in glia and found that the cells survived and differentiated into astrocytes in the spinal cord, as well as improved motor function and survival [181].

In addition to using glial cells as a transplant therapy, human iPSCs from ALS patients and healthy controls were differentiated to astrocyte progenitors and injected into the spinal cord of ~2-month-old severe combined immunodeficient (SCID) mice [186]. The cells were assessed 9 months post-transplant and found to be mostly positive for GFAP as well as being larger and possessing more processes (compared to the endogenous mouse astrocytes), and these astrocytes contacted the endogenous blood vessels and surrounded neurons. The authors studied whether the astrocytes differentiated from patient cells versus non-ALS cells differed when transplanted to the mouse spinal cord. Astrocytes from sporadic ALS patients showed characteristics of being more reactive and having more pathological aggregates compared to the non-ALS transplanted astrocytes. Additionally, the mice transplanted with the patient cells lost motor neurons (preceded by loss of non-motor neurons) compared to the healthy cell transplanted mice and showed motor impairments in grip strength and gait. This study demonstrates the importance of the origin of the cells used for the transplant and a model such as this is useful to further study mechanism of how these cells’ endogenous properties lead them to develop disease.

Studies are now starting to focus on using microglia progenitors differentiated from iPSCs. Microglial activation (or reactive microgliosis) is a common feature of not only acute brain injury but neurodegenerative diseases as well (Table 1). Whether activation of microglia in these diseases is a cause or a consequence of protein aggregation or neuronal dysfunction/death remains to be elucidated, making it a central question across fields. As microglia have been shown to interact with the abnormal aggregates often present in many neurodegenerative diseases [205] and regulate neurogenesis [206], both the underlying mechanism of microglia in neurodegenerative disease as well as their utility as therapy are incredibly pertinent.

Studying microglia reactivity in vitro as discussed in previous sections can be useful; however, it comes with the caveat that these cells are susceptible to their environment [207]. Therefore, transplantation may incur the advantage of having the whole brain environment. Human iPSCs differentiated into microglia precursors, as evidenced by expression of CD11b and CD45, were transplanted to the lateral ventricles of transgenic immunodeficient neonatal mice that also carry human transgenes for CSF1, IL3, KITL, and CSF2 [208]. These mice were used since their immunodeficiency, combined with a host environment that favours human immune cells, are ideal for transplantation of microglia. The precursors were shown to turn into mature microglia: at 2 months post-transplantation the cells, located in the striatum and cortex, were positive for P2RY12, Iba1, and TMEM119, as well as becoming more morphologically distinct. The authors also compared how the microglia fared in the rodent brain versus in culture. They found that the microglia transplanted to the brain resembled primary human microglia more closely in gene expression, whereas microglia that remained in the dish more closely mimicked a disease state. Additionally, when the mice that received the transplanted microglia were stimulated with LPS, the cells took on a more “activated” state. This study demonstrated that it is possible to transplant microglial progenitors to the mouse brain and that these develop into mature microglia that are more similar to human microglia. Another study showed similar results [209]. The authors also transplanted microglia precursors derived from human iPSCs to postnatal day 0 mice (immunodeficient and expressing human CSF1); in this case, they were injected above and into the hippocampus. At 6 months post-transplantation, mature microglia cells expressing TMEM119 and P2RY12 and with longer processes and more complex morphology, were found throughout the mouse brain. Examining the functionality of these cells showed that they pruned synapses, contacted blood vessels, and phagocytosed oligodendrocytes—this was evident from 3 weeks up until 6 months post-transplantation. A thorough comparison of gene expression patterns of these microglia was also performed, and similarly to the above study, the cells showed strong resemblance to adult human microglia. Interestingly, the gene expression profile of these microglia revealed that they express human neurodegenerative disease-relevant genes differentially to mouse microglia: MS, AD, and PD genes were more highly expressed. Lastly, the authors tested whether the cells would respond to demyelination and found upregulated expression of genes also observed in MS patients. The success of these studies is an important proof-of-concept in transplantation of immature microglia to the brains of neonatal mice.

In relation to neurodegenerative diseases, one study has transplanted human iPSC-derived microglia to an AD mouse model. In 2019, Hasselmann and colleagues [185] transplanted microglia progenitors to postnatal day 1 humanized immunodeficient mice as in the above-mentioned studies. These also differentiated into mature microglia, resembled human microglia in their transcriptomic profile, and became activated after injection of LPS, as above. Further, the microglial cells took on different morphologies depending on their brain location, and functional studies showed that they were actively surveying the environment, responding to acute injury via extension of processes, as well as phagocytosing debris of degenerating neurons. With the success of these experiments, the authors expanded the studies by using a genetic AD mouse (the 5xFAD model, which has five familial mutations of AD [210]) crossed with humanized immunodeficient mice in order to study how the transplanted human microglia respond to amyloid plaques. Importantly, the microglia precursors were injected bilaterally to the cortex and hippocampus of adult (3-month-old) mice and aged for 9 months. The microglial response to Aβ was characterized by downregulation of P2RY12, responsible for microglia chemotaxis, upregulation of markers associated with the microglial response to disease: APOE, CD9, CD11C, MERTK, and TREM2, as well as becoming amoeboid in shape and in some cases phagocytosing the fibrillar form of the protein. The transcriptomic analysis also revealed a differential gene expression profile that was specific to the human microglia response to Aβ. The authors then took two examples to perform immunofluorescence staining with and compared this to brain sections from human AD patients. They found that the expression of these two genes in the transplanted microglia was similar to that of the endogenous microglia staining pattern in the patient brain. This study clearly showed that the transplantation of microglia derived from human iPSCs to a mouse model of neurodegenerative disease has the potential to give insight into the human condition.

## 5. Conclusions

Using iPSCs to understand glial cell involvement in human neurodegenerative diseases, including AD and PD where they are heavily implicated in mechanism, will continue to be crucial for future research. The advent of 3D brain organoids derived from iPSCs has also become a major area of research in recent years, since modelling the brain microenvironment is necessary to understand the complexities of human disease. This will be particularly important for glia as these cells interact with neurons and other CNS components such as the BBB to achieve a fully functioning system. In general, it is clear that human-derived cells are important for studying neurodegenerative disorders, which cannot be modelled with complete accuracy in animals alone. The next logical step has, therefore, been transplanting differentiated iPSCs directly into the brains of animals. Since glial cells are sensitive to their environment, transplantation to the living brain may be important in further studying how they contribute to disease pathogenesis. The ability of these grafted cells to take on a more human-like disease state when transplanted to the rodent brain is a promising way forward to elucidate mechanism of neurodegenerative diseases, for which the causes are still unknown. Further, if glial cells become dysfunctional in neurodegenerative disease and contribute to disease pathology, replacing them could be utilised as a future therapy.

These three ways of modelling disease have also given researchers further information in regard to how much human cells differ from rodent cells, from gene expression to function. By studying single or particular populations of iPSC-derived cells taken from the dish, or isolated from organoids or rodent brain, we can begin to gain knowledge on how these cells may change their gene expression in response to disease. Additionally, their response to both acute pathology and long-term function can be studied over time, the latter of which is particularly important in neurodegenerative disease. Since cells derived from animals may not fully recapitulate key features of diseases that are only observed in humans, using cells derived from human tissue without the associated ethical issues or limitations on the amount is an incredibly useful research tool.

With glial cells making up approximately half of the cells in the CNS, it is surprising that they have only relatively recently received more attention. Astrocytes, microglia, and oligodendrocytes have been shown to not only interact with neurons and the surrounding environment, but each other as well. Therefore, future research will need to focus on not just individual cell types, but on the intricate interplay between all of the cells in the brain in order to elucidate the mechanisms of neurodegenerative diseases. As we are still only beginning to understand how each type of glial cell contributes to major neurodegenerative diseases, researchers will also need to delve deeper into how these cells become dysfunctional in order to find future therapies. Glia are clearly involved in the development of the CNS as well as functioning as critical support cells for neurons. Many neurodegenerative diseases have the common property that neurons are lost in a particular region, and it is often still unclear why that area is vulnerable to cell death while others are not. With the vast roles of glia in regulating cell growth, maturation, pruning, and also providing metabolic and trophic support, it is logical that their potential dysfunction can fundamentally affect neuron survival and proper functioning. Additionally, astrocytes and microglia become reactive and likely overactive in a disease state, and this should continue to be a primary research focus, as this is also occurring in many diseases.

Another important aspect of glial cells, though out of the scope of this review, is that during development they can act as neural stem cells or progenitors of other types of glia. In most injury cases, once a neuron dies it is not regenerated. However, surrounding glia at the site of injury, particularly reactive astrocytes, may provide stem and progenitor cells that can be directed towards neuronal fate (this concept reviewed in [211]). Though reprogramming these cells in the living brains of mammals is complicated, involving viral methods to direct these cells to neurons, provision of trophic support, and ensuring that they integrate properly to the network, it has been achieved (reviewed in [212]). This technique shows promise in that it bypasses the issue of immune rejection as the patient’s own cells already present in the brain are utilised.

In conclusion, two major aspects are evident: glia are important when it comes to neurodegenerative disease mechanism and having a sustainable pool of cells derived from both healthy human subjects and diseased patients gives researchers a valuable tool to study these cells in human disease. Though models alone are not a silver bullet to cure neurodegenerative diseases, they can give us much-needed knowledge to bring us closer to a future therapy.

## Figures and Tables

**Figure 1:** The cells of the central nervous system (CNS). Neurons (yellow) are at the core of the CNS, and their primary function is to deliver neuronal signals. The different glial cells—astrocytes (green), oligodendrocytes (pink), and microglia (blue)—support neuronal function.

**Figure 2:** Induced pluripotent stem cells (iPSCs) can be used to create a variety of different cell types, including astrocytes, microglia, and oligodendrocytes.

**Figure 3:** Left side: iPSC-derived brain organoids from a healthy human subject can be used to specifically model the brain microenvironment, including studying interactions between a variety of cell types. Additionally, modifications such as integration of microglia and endothelial cells provides opportunities to further elucidate functions of these cells in vitro. Right side: Using brain organoids derived from the cells of a human patient is a powerful tool to study disease mechanisms. Typical features of neurodegenerative diseases can be modelled in brain organoids, namely plaque formation, glia activation, and neuronal dysfunction. BBB=blood–brain barrier.

**Figure 4:** In animal models using iPSCs, progenitor cells are derived from a patient’s somatic cells and differentiated to neuronal or glial precursors. These cells are then transplanted to the rodent brain and studied in situ in order to make a humanized model of disease.

**Table 1:** Table of the most common neurodegenerative diseases with their major properties and how glial cells are involved in each disease.

Disease	Known Mutations	Pathological Protein	Common Symptoms	Astrocyte Involvement	Microglia Involvement	Oligodendrocyte Involvement
Alzheimer’s disease	*APP, PSEN1, PSEN2,* *APOEε4* allele (risk factor)	Amyloid-β, tau	Memory impairment, disorientation, delirium and dementia	Reactive astrocytes ↑, neuroprotection ↓, synaptogenesis ↓, altered phagocytosis [56,57,58,59,60]	Microgliosis ↑ [57,59,61,62,63]	Differentiation ↓, death ↑, oligodendrocyte size ↓, myelinating oligodendrocytes ↓ [59,64]
Amyotrophic lateral sclerosis	*SOD1, C9ORF72, FUS, TARDBP, VAPB, FIG4, OPTN, VCP, SQSTM1/p62, SIGMAR1, UBQLN2, TBK1, PDIA1, PDIA3, CCNF*	TDP-43	Progressive weakness of muscles, spasticity, difficulties in speaking, breathing and swallowing, fatal	Reactive astrogliosis ↑, neuroprotection ↓, synaptogenesis ↓, phagocytosis ↓ [17,56,65,66]	Microglial activation ↑ (cross-talk between both astrocytes and oligodendrocytes), secretion of toxic factors ↑ [17,65,67,68]	Progenitor cell NG2+ proliferation ↑, abnormal morphology ↑, neurotoxic interactions ↑, differentiation ↓, death ↑ [69,70]
Creutzfeld–Jacob disease	*PRNP*; several mutations, e.g., *P102L, P105L, D178N, V180I, E200K, V203I*	Prion protein	Dementia, amnesia, personality changes, fatal	Reactive astrocytes ↑, emperipolesis (oligodendrocyte engulfment) [71,72,73,74,75,76]	Reactive microglia↑ [71,75,77]	Interaction with reactive astrocytes, emperipolesis (astrocytes engulf oligodendrocytes) [72,74]
Huntington’s disease	*HTT*	huntingtin	Abnormal involuntary movements, psychiatric symptoms, cognitive decline	Reactive astrogliosis ↑, neuroprotection ↓, synaptogenesis ↓, phagocytosis ↓ [15,56,78,79,80]	Microgliosis↑, phagocytosis ↑ [15,79,81]	Remyelination ↓, differentiation ↓, death ↑ [82,83,84]
Parkinson’s disease	*PARK* mutations; *LRRK2, PARK2 PARK7, PINK1, SNCA*	α-synuclein	Rigidity, tremor, fatigue, depression, pain, and cognitive problems	Reactive astrocytes ↑: neuroprotection ↓, synaptogenesis ↓, phagocytosis ↓, Ca^2+^ release from ER ↑, mitochondrial function ↓, mitochondrial respiration ↓, α-synuclein clearance ↓ [56,85,86,87]	Reactive microgliosis↑, phagocytosis ↑, proinflammatory cytokines ↑ [86,88,89,90]	Differentiation ↓, death ↑ [91]
Spino- cerebellar ataxia	group of ~30 diseases, e.g., *SCA1, SCA2, TMEM240, TGM6*	expanded polyQ peptides	Balance impairment, coordination problems, speech impediment, can be fatal	Reactive astrogliosis ↑, proinflammatory cytokines ↑ [92,93]	Reactive microgliosis ↑, release of proinflammatory cytokines ↑ [92]	Demyelination ↑ (toxic gain of function mutation) [94]
Spinal muscular atrophy	*SMN1, SMN2, TRPV4, UBA1, DYNC1H1, PLEKHG5, IGHMBP2, GARS, FBXO38*	SMN protein depletion	Muscle weakness, muscle atrophy, fasciculations, impaired speaking, breathing, swallowing, and walking, (childhood form) fatal	Reactive astrogliosis ↑, proinflammatory cytokines ↑, basal Ca^2+^↑, ATP stimulation response↓, Notch signaling dysregulation ↑ [95,96,97]	Reactive microgliosis, proinflammatory cytokines ↑, suspected synaptic stripping caused by enhanced phagocytosis [95,96]	Differentiation ↓, dysfunction ↑, precursor cell proliferation ↓ [96,98]

↑ = increased; ↓ = decreased.

**Table 2:** Table of preclinical transplant studies performed in rodents using human-derived induced pluripotent stem cells (iPSCs) in neurodegenerative diseases, both as a therapy and to model disease.

Transplant as Therapy							
Disease	Cell Source	Cell Type	Model	Injection Site	Post-Transplantation Follow-Up Time	Outcomes	Reference
PD	Sporadic patients	DA neurons	6-OHDA rats	Striatum	16 weeks	Motor asymmetry reduced	[173]
AD	Human cell line	Cholinergic neurons	Transgenic *APP* mice	HPC	45 days	Improved spatial memory	[179]
ALS	Healthy humans	Motor neurons	Transgenic *SOD1* mice	Systemic and intrathecal	50 days	Improved motor behaviour and survival	[180]
ALS	Human cell line	Astrocytes	Transgenic *SOD1* mice	Spinal cord	40 days	Improved motor behaviour and survival	[181]
HD	Juvenile patients	GABAergic neurons	Quinolinic acid rats	Striatum	12 weeks	Behavioural improvement	[182]
**Transplant as Model**							
**Disease**	**Cell Source**	**Cell Type**	**Mouse**	**Injection Site**	**Post-Transplantation Follow-Up Time**	**Outcomes**	**Reference**
AD	FTD patient	Cortical neurons	Neonatal ID *APP*/*PSEN1* mutant	Frontal cortex	8 months	AD pathology in transplanted neurons	[183]
AD	AD patient	Excitatory and inhibitory neurons	Adult *APOEε3* or *APOEε4* transgenic	HPC	7 months	AD phenotype in neurons	[184]
AD	Human cell lines	Microglia	Adult humanized ID 5xFAD transgenic	Cortex, HPC	9 months	AD phenotype in microglia	[185]
ALS	ALS patients and healthy controls	Astrocytes	Adult SCID mice	Spinal cord	9 months	Loss of motor neurons, motor deficits	[186]

Abbreviations: 5XFAD = 5 familial Alzheimer’s disease mutations; 6-OHDA = 6-hydroxydopamine; AD = Alzheimer’s disease; ALS = amyotrophic lateral sclerosis; APP = amyloid precursor protein; DA = dopamine; FTD = frontotemporal dementia; HD = Huntington’s disease; HPC = hippocampus; ID = immunodeficient; PD = Parkinson’s disease; PSEN1 = presenilin 1; SCID = severe combined immunodeficient; SOD1 = superoxide dismutase 1.
